# DL-3-N-Butylphthalide Promotes Cartilage Extracellular Matrix Synthesis and Inhibits Osteoarthritis Development by Regulating FoxO3a

**DOI:** 10.1155/2022/9468040

**Published:** 2022-07-20

**Authors:** Yaxin Zhang, Jihang Dai, Lianqi Yan, Qun Lin, Haixiang Miao, Xingkai Wang, Jingcheng Wang, Yu Sun

**Affiliations:** ^1^Dalian Medical University, Dalian 116044, China; ^2^Department of Orthopedics, Northern Jiangsu People's Hospital Affiliated to Yangzhou University, Yangzhou 225000, China

## Abstract

Osteoarthritis (OA) has been reported as a progressive disease in the elderly, primarily characterized by degenerated articular cartilage. There has been no satisfactory drug for the treatment of OA. DL-3-n-butylphthalide (NBP), a small molecule compound extracted from celery seeds, may have antiapoptotic, antioxidant, and anti-inflammatory activities in numerous studies. However, the effects of NBP on OA and its mechanisms have been rarely reported. In this study, the effect of NBP on OA in vitro and in vivo and its possible mechanism were investigated. The results showed that NBP injection into the knee joint inhibited osteoarthritis development in a rat model of osteoarthritis induced by DMM+ACLT. NBP could increase the expressions of extracellular matrix-related components (such as type II collagen, aggrecan, proteoglycan 4, and SRY-box 9) in human osteoarthritic chondrocytes and cartilage explants. Moreover, NBP promoted the expressions of SOD and CAT. NBP upregulated the expression of FoxO3a by inhibiting the PI3K/AKT pathway, which subsequently inhibited the apoptosis of human OA chondrocytes. In conclusion, NBP promotes cartilage extracellular matrix synthesis and inhibits osteoarthritis development and the underlying mechanism related to the activation of FoxO3a.

## 1. Introduction

Osteoarthritis (OA) is a chronic degenerative joint disease and characterized by cartilage destruction, subchondral bone sclerosis, synovial inflammation, and osteophyte formation [1]. OA has been reported as the main cause of pain and disability among the elderly worldwide, which resulted in a serious effect on their quality of life and health [2, 3]. The major strategies for early OA are anti-inflammatory and analgesic treatment [4]. However, the existing drugs are only capable of relieving pain while having no significant clinical effect on the prevention or improvement of OA diseases.

Articular cartilage is an avascular tissue that consists of chondrocytes and their extracellular matrix (ECM). ECM maintains the mechanical properties of articular cartilage and the function of joint lubrication [5, 6]. Chondrocytes, the only resident cells in the cartilage have been found to play vital roles in regulating the synthesis of ECM and maintaining the structure of cartilage [7, 8]. Therefore, the status of chondrocytes has a direct effect on the function of articular cartilage.

Dysregulation of apoptosis can result in pathological conditions in the body, such as cancer, dysplasia, and degenerative diseases [9]. Existing studies confirmed that chondrocyte apoptosis has a significant correlation with the destruction of articular cartilage and matrix degradation, showing a positive correlation with the severity of OA [10, 11]. Moreover, oxidative stress plays an important role in the occurrence and development of OA. Excessive production of reactive oxygen species in articular cartilage induces oxidative damage to chondrocytes. This leads to chondrocyte apoptosis and ECM degradation, which causes irreversible damage to articular cartilage. Therefore, drugs regulating apoptosis and oxidative stress may serve as potential therapeutic approaches for the treatment of OA.

Among the Forkhead box O (FoxO) subfamilies, FoxO3a plays a key role in oxidative stress, apoptosis, proliferation, and deoxyribonucleic acid (DNA) damage. Several studies demonstrated that upregulating FoxO3a or inhibiting its degradation could inhibit apoptosis in cells [12, 13]. TRIM33 protects osteoblasts from oxidative stress-induced apoptosis by inhibiting the ubiquitination and degradation of FoxO3a [13].

DL-3-n-Butylphthalide (NBP) refers to a small molecule compound extracted from celery seeds. Thus far, a considerable number of studies have found that NBP has broad therapeutic benefits and plays a vital role in many neurodegenerative diseases [14, 15]. In general, its mechanism primarily consists of antiapoptosis, antioxidation, anti-inflammation, and proangiogenesis [16, 17]. NBP has been shown to have antiapoptotic effects in a variety of cells, including neuronal cells, cardiomyocytes, and bone marrow stem cells [18–20]. However, no relevant report has been conducted on the protective and therapeutic effects of NBP on osteoarthritis due to the multitarget therapeutic properties of NBP.

This study is aimed at investigating the effect of NBP on the ECM components (such as type II collagen (COL2A1), aggrecan (ACAN), proteoglycan 4 (PRG4), and SRY-box 9 (SOX9)) synthesis and at verifying the protective effect by inhibiting OA development in rats, and the relevant molecular mechanisms were explored.

## 2. Materials and Methods

### 2.1. Reagents

NBP (purity ≥99%) was provided by MedChemExpress (Shanghai, China). HE, safranin O-fast green, and alcian blue staining solutions originated from Solarbio (Wuhan, China). Cell-Counting Kit-8 (CCK-8) was purchased from Dojindo (Kumano, Japan). TRIzol reagent, dimethyl sulfoxide (DMSO), and immunohistochemical staining kit were purchased from Absin (Shanghai, China). Penicillin, streptomycin, 0.25% trypsin, type II collagenase, fetal bovine serum (FBS), and Dulbecco's modified Eagle medium (DMEM) were provided by Gibco (NY, USA).

### 2.2. Human OA Chondrocytes Isolation and Culture

Human OA chondrocytes were collected from patients receiving total knee replacement for osteoarthritis in accordance with the regulations of the Ethics Committee of Northern Jiangsu People's Hospital. In brief, the cartilage pieces were washed, cut into small pieces, and then digested in 0.25% trypsin for 30 min at 37°C. After the trypsin was removed, the tissue was digested with 0.2% type II collagenase for 6 h at 37°C. The cells were filtered and then collected into DMEM/F12 medium containing 10% FBS. Next, the cells were cultured using a humidified incubator with 5% CO_2_ at 37°C.

### 2.3. Cell Viability

The effect of NBP on chondrocyte viability was measured using the CCK8 kit. Firstly, the chondrocytes (5000 cells/well) were seeded into 96-well plates and incubated for 24 h. Subsequently, the chondrocytes were incubated with NBP at different concentrations (0.01, 0.1, 1, 10, and 100 *μ*M) for 24 h. Next, 10 *μ*L CCK8 solution was added into each well and incubated for 2 h. Lastly, the absorbance was measured at 450 nm using a microplate reader.

### 2.4. qRT-PCR Analysis

The total RNA was extracted using the TRIzol reagent. cDNA was synthesized from purified RNA (1 *μ*g) using HiScript III RT SuperMix for qPCR kit. Quantitative real-time PCR (qRT-PCR) was performed using the Applied Biosystems StepOnePlus Real-Time PCR System (Foster City, CA, USA). The amplification conditions included 5 min at 95°C followed by 40 cycles of 10 sec at 95°C and 30 sec at 60°C, 15 sec at 95°C, 60 sec at 60°C, and 15 sec at 95°C for the melt curve. The target mRNA was standardized at GAPDH level. Information regarding the primer sequences is shown in Table 1.

### 2.5. Western Blotting

The drug-treated chondrocytes were lysed using a mixture of radio immunoprecipitation assay (RIPA) lysis buffer and protease inhibitor cocktail. The proteins with equal amounts (30 *μ*g) were separated on the sodium dodecyl sulfate polyacrylamide gel electrophoresis (SDS-PAGE) gel and then transferred to a polyvinylidene fluoride (PVDF) membrane. After being blocked with 5% bovine serum albumin for 1 h, the membranes were incubated with the primary antibodies overnight at 4°C. Subsequently, the membranes were incubated with the secondary antibodies for 1 h at ambient temperature. Lastly, the membranes were visualized using the BIO-RAD ChemiDoc XRS+system. The primary antibodies consisted of COL2A1 (Bioss, 1 : 1000), ACAN (Bioss, 1 : 1000), FoxO1 (CST, 1 : 1000), FoxO3a (CST, 1 : 1000), p-FoxO3a (CST, 1 : 1000), FoxO4 (CST, 1 : 1000), PI3K (CST, 1 : 1000), p-PI3K (CST, 1 : 1000), AKT (CST, 1 : 1000), p-AKT (CST, 1 : 1000), Bax (CST, 1 : 1000), Bcl-2 (CST, 1 : 1000), Caspase 3 (CST, 1 : 1000), SOD2 (ABclonal, 1 : 1000), CAT (ABclonal, 1 : 1000), GAPDH (CST, 1 : 1000), and *β*-actin (CST, 1 : 1000).

### 2.6. Immunofluorescence

The human OA chondrocytes were seeded on the cover slips in 6-well plates and then incubated for 24 h with or without NBP (0.1 *μ*M). Next, the cells were rinsed in PBS and then fixed with 4% paraformaldehyde. Subsequently, the cells were permeabilized with 0.1% Triton X-100 and blocked with 5% bovine serum albumin. Furthermore, the cells were incubated with the primary antibodies against type II collagen (COLII, Abcam, 1 : 200), ACAN (Bioss, 1 : 100), and FoxO3a at 4°C overnight. Afterward, the cells were incubated with FITC conjugated anti-rabbit IgG (Abcam, 1 : 1000) or anti-mouse IgG (Abcam, 1 : 1000) for 1 h in the dark. The nuclei were stained with DAPI (Beyotime, China). Lastly, the cover slips were observed under a fluorescence microscope.

### 2.7. TUNEL Analysis

The apoptosis of chondrocytes was detected using the TUNEL BrightGreen Apoptosis Detection Kit (Vazyme, China). The human chondrocytes were seeded on the 6-well plate coverslips and then treated with NBP at different concentrations for 24 h. Subsequently, the chondrocytes were fixed with 4% paraformaldehyde for 25 min, and the permeability of chondrocytes and their nuclear membranes increased using 0.2% Triton X-100. The chondrocytes were incubated with 50 *μ*L of TUNEL reaction mixture with terminal deoxynucleotidyl transferase (TdT) for 1 h at 37°C in accordance with the manufacturer's instructions. The nuclei of chondrocytes were stained with DAPI. The TUNEL-positive cells were observed and detected under the fluorescence microscope.

### 2.8. Flow Cytometry Analysis of Chondrocytes Apoptosis

The apoptosis of the chondrocytes was detected using the Annexin V-FITC/PI Apoptosis Detection Kit (Beyotime, China). The human chondrocytes treated with NBP at different concentrations were collected and then washed with precooled PBS 3 times. Subsequently, the chondrocytes were resuspended with 195 *μ*L Annexin V-FITC binding buffer. Afterward, 5 *μ*L Annexin V-FITC and 10 *μ*L PI staining were introduced into the solution, respectively, for 20 min at ambient temperature in the dark. Flow cytometry (BD Biosciences) was used to count the apoptotic cells.

### 2.9. Detection of Oxidative Stress Levels in Chondrocytes

The human OA chondrocytes were treated with NBP at different concentrations for 24 h and then washed with pre-cooled PBS 3 times. Afterwards, the cells were collected and centrifuged. The expression levels of superoxide dismutase (SOD) and glutathione (GSH) were detected using Total Superoxide Dismutase Assay Kit (Beyotime, China) and GSH Assay Kit (Beyotime, China), respectively.

### 2.10. Culture of Human OA Cartilage Explants

The cartilage explants from the patients of total knee replacement were taken and then cut into pieces of approximately 1 mm^3^. The explants were evenly separated into DMEM containing 10% FBS, with or without NBP (0.01, 0.1, 1 *μ*M), respectively. The solution was changed every 3 d. The explants were collected after 2 weeks for histological analysis as well as the detection of mRNA expression levels, DNA, and glycosaminoglycan (GAG).

### 2.11. Biochemical Assays of Cartilage Explants

The cartilage explants were digested in a solution of papain (containing 125 mg/mL papain, 5 mM cysteine HCl, and 5 mM EDTA in PBS) at 60°C for 12 h. The GAG content was assessed using the DMMB COLORIMETRY kit (GENMED, China). Furthermore, the DNA content was assessed using the dsDNA HS Assay Kit for Qubit (Yeasen, Shanghai, China). 10 *μ*L of lysate was mixed with 190 *μ*L of the test solution and then incubated for 2 min in the dark.

### 2.12. Establishment of OA Model and Intra-articular Injection of NBP

30 male SD rats weighing 200 g were provided by the Comparative Medicine Center of Yangzhou University. All animal experiments gained the approval from the Animal Care and Use Committee of Yangzhou University. The rat OA model was built by destroying the medial meniscus (DMM) and the anterior cruciate ligament (ACL). The rats were anesthetized through the intraperitoneal injection of pentobarbital. The DMM+ACLT of the right knee was destroyed, and the left knee joint received an arthrotomy as a sham operation group. All rats randomly fell into five groups, including the control group (sham operation), the vehicle group (saline group), and the NBP treatment group (30, 60, and 90 mg/kg). The rats were injected 100 *μ*L of NBP or saline into the knee joints of twice a week for 8 weeks.

### 2.13. Histological Analysis

After the rats were euthanized, the intact knee joints were removed and fixed with 4% paraformaldehyde for 48 h. The knee joints were then decalcified in EDTA solution for 1 month and embedded in paraffin for serial sections. The sections were stained with hematoxylin-eosin (HE) and safranin O-fast green to assess the degree of cartilage destruction. The severity of OA was evaluated based on the Osteoarthritis Research Society International (OARSI) scoring system [21].

### 2.14. Analgesic Experiments of Plate Method

In brief, the hot plate apparatus was heated to 55°C. The hind limbs of the rats were attached onto the hot plate, and the reaction time was recorded when the rats' feet were licking and twitching. If the hind limb reaction time was longer than 30 s, the rat was removed immediately to avoid scalding. The respective rat was measured 3 times.

### 2.15. Static Load Test

The rats were placed in a bipedal balance pain tester (BIO-SWB-R), and their hind limbs were placed onto two separate sensor plates. The duration of static load test was set to 9 sec. The weight difference between the left hind limb (sham operation) and right hind limb (operation) was recorded. The measurements were repeated 3 times for the respective rat.

### 2.16. Network Pharmacology

In brief, the 2D and 3D chemical structures of NBP were obtained from PubChem database (https://pubchem.ncbi.nlm.nih.gov/) and then saved in an SDF format. The potential targets were predicted using Pharmmapper (http://lilab-ecust.cn/pharmmapper/). OA disease genes were collected from the OMIM (http://omim.org/) and Genecards (http://www.genecards.org) databases. The OA-related gene sets were acquired by merging and deduplicating the search results of Genecards and OMIM. A comparison between the potential target set of NBP and the target set of OA was drawn, and the overlapped part of the two was considered the target of NBP for OA treatment. The intersection was investigated using the R language for gene ontology (GO) enrichment analysis and Kyoto Encyclopedia of Genes and Genomes (KEGG) pathway enrichment analysis.

### 2.17. RNA Sequencing of Chondrocyte Transcriptome

The total RNA was extracted from the chondrocytes administrated with or without NBP (0.1 *μ*M) using Trizol reagent. The obtained RNA samples were sent to APPLIED PROTEIN TECHNOLOGY (Shanghai, China) for RNA sequencing. The expression FPKM value of the respective gene in each sample was determined using featureCounts software. The differentially expressed genes were counted using the DESeq algorithm. The genes with significantly different expressions were identified as follows: |log2foldchange| > 1 and *P* < 0.05. Through the GO analysis, the biological functions of differential genes were described, which included biological processes (BP), molecular function (MF), and cellular components (CC). The pathways with significant enrichment of differential genes were described by KEGG database analysis.

### 2.18. Lentiviral Constructions and Infection

The lentiviral construct in this paper originated from GENECHEM (Shanghai, China). The hU6-MCS-CBh-gcGFP-IRES-puromycin lentiviral recombinant vector was established as the siFoxO3a (knockout FoxO3a) virus. The sequence of siFoxO3a employed included TTCCTTGCTCATATCCCATAT. The chondrocytes were seeded in the 6-well plates; when these chondrocytes had 60% confluence, they were infected with FoxO3a knockdown lentivirus. After puromycin (0.75 *μ*g/mL) was used for selection for three days, a stable strain was generated. Fluorescence signal was observed under the microscope. FoxO3a expression was assessed using qRT-PCR and Western blot assay.

### 2.19. Statistical Analysis

For at least three separate determinations per group, the data are expressed as mean ± standard deviation (SD). The statistical significance of difference between groups was determined through Student's *t*-tests and one-way analysis. When *P* < 0.05, the difference was considered with statistical significance.

## 3. Results

### 3.1. Identification of Human OA Chondrocytes

The extracted cells were confirmed as chondrocytes by alcian blue staining and immunofluorescence staining. The proteoglycan in chondrocytes was stained blue with alcian blue staining solution, and COLII was stained red by immunofluorescence (Figures 1(b) and 1(c)). As indicated by both staining results, the extracted cells were human OA chondrocytes.

### 3.2. NBP Increased ECM Anabolism of Human OA Chondrocytes

To verify whether the effect of NBP on the ECM synthesis of chondrocytes, cells were treated with different concentration of NBP for 24 h. The chemical structure of NBP is shown in Figure 1(a). CCK-8 assay indicated that NBP had no inhibitory effect on the viability of chondrocytes at 0-10 *μ*M concentrations (Figure 1(d)). After being treated with NBP (0.01-10 *μ*M), Western blot assay demonstrated that the protein expressions of COL2A1 and ACAN was significantly increased (Figures 1(e) and 1(f)). The mRNA levels of ECM-related genes including COL2A1, ACAN, PRG4, and SOX9 were upregulated after NBP treatment (Figure 1(g)). 0.1 *μ*M NBP significantly increased the expressions of COL2A1, ACAN, and SOX9 compared with those of other groups. Moreover, COLII and ACAN proteins were significantly upregulated after treated with 0.1 *μ*M NBP by the immunofluorescence (Figures 1(h) and 1(i)). These results demonstrated that NBP could increase ECM anabolism of human OA chondrocytes.

### 3.3. NBP Promoted ECM Anabolism in OA Cartilage Explants

To study whether NBP promoted ECM anabolism in cartilage explants, human OA cartilage explants were cultured for 2 w in the presence or absence of NBP treatment. The safranin O-fast green staining showed that proteoglycan content in NBP-treated group significantly increased compared with that in the vehicle group. The increase of proteoglycan content and the average optical density (AOD) value was the most significant at 0.1 *μ*M (Figures 2(a) and 2(c)). The result of immunohistochemistry staining demonstrated that NBP significantly promoted the expression of COLII after NBP treatment for 2 w (Figure 2(b)). The quantitative analysis indicated that NBP increased the GAG content and DNA content in OA cartilage explants (Figures 2(d) and 2(e)).

Moreover, the mRNA expression levels of ECM-related components after the NBP treatment were performed by qRT-PCR. The mRNA levels of COL2A1, ACAN, PRG4, and SOX9 in cartilage explants after being treated with NBP (0.1 *μ*M) significantly increased compared with those in the vehicle group (Figures 2(f)–2(i)). Therefore, NBP could increase synthesis of ECM-related components and promote ECM anabolism in OA cartilage explants.

### 3.4. NBP Inhibited the Development of Knee OA in the DMM+ACLT Rat Model

To determine the protective effect of NBP on OA development, the rat model of knee OA was built by DMM+ACLT surgery. The intraknee injections of NBP or vehicle alone (saline) were performed in rats twice a week for 8 weeks. As indicated by HE and safranin O-fast green staining, superficial cartilage destruction, cartilage erosion, and proteoglycan loss were obviously found in the vehicle group. However, there was significant improvement in superficial cartilage destruction, cartilage erosion, and proteoglycan loss in the NBP-treated group compared with those in the vehicle group, and 60 mg/kg NBP had a significant effect (Figure 3(a)). NBP significantly promoted the expression of COLII compared with the vehicle group from the immunohistochemistry result (Figure 3(a)). The OARSI score of the rats in the NBP group was significantly lower than that in the vehicle group (Figure 3(b)). Moreover, the hot plate test was used to measure the reaction time to heat and the static load test was used to detect the difference in weight bearing of lower limbs, both of which could reflect pain of knee joint and indirectly evaluate the degree of OA in rats. The hot plate and static load tests showed that intra-articular injections of NBP could significantly alleviate the pain caused by OA in rats (Figures 3(c) and 3(d)). The above results showed that NBP could inhibit the development of knee OA in the DMM+ACLT rat model and 60 mg/kg NBP exerted significant effect.

### 3.5. NBP Inhibited Apoptosis and Oxidative Stress of Human OA Chondrocytes

The effects of NBP on apoptosis and oxidative stress of human OA chondrocytes were detected after treated with NBP at different concentrations for 24 h. The flow cytometry analysis and TUNEL staining showed that the apoptosis rate and TUNEL positive cells significantly decreased after NBP treatment compared with that in vehicle group, indicating that NBP could inhibit chondrocytes apoptosis (Figures 4(a)–4(d)). Moreover, the expressions of apoptosis-related factors were measured using qRT-PCR and Western blot assay. NBP treatment inhibited the mRNA and protein expressions of Bax and Caspase 3 and increased expression of Bcl-2 (Figures 4(e)–4(g)). These results demonstrated that NBP inhibited apoptosis of human OA chondrocytes.

Intracellular reactive oxygen species (ROS) scavenging enzymes such as SOD, GSH, and catalase (CAT) were usually used as biomarkers to evaluate the level of cellular oxidative stress. After treatment with NBP, the expression levels of SOD, GSH, and CAT significantly increased in human OA chondrocytes compared with the untreated group (Figures 4(g)–4(k)). The results indicated that NBP could suppress the level of oxidative stress of human OA chondrocytes by increasing the expression of ROS scavenging enzymes.

### 3.6. Bioinformatics Analysis Based on Network Pharmacology of NBP on OA

A total of 211 potential targets of NBP and 3114 OA genes were selected. Among these targets, there was 108 common targets considered as potential targets for NBP in treating OA (Figure 5(a)). The 108 common targets were investigated by GO term for functional enrichment, and the results demonstrated collagen-containing extracellular matrix (Figure 5(b)). The KEGG enrichment analysis from top 20 significantly-related pathways demonstrated that PI3K-AKT signaling pathway, apoptosis, and FoxO signaling pathway were enriched (Figure 5(c)). These results of bioinformatics analysis of network pharmacology supported the positive effect of NBP in the treatment of OA.

### 3.7. Analysis of Transcriptome Sequencing after NBP Treatment

To clarify targets of NBP on treating OA, transcriptome sequencing was performed on human OA chondrocytes after treated with NBP (0.1 *μ*M) for 24 h. Among differentially expressed genes in the transcriptome, FoxO3a was significantly upregulated (Figure 5(d)). GO analysis for examine candidate genes demonstrated that extracellular matrix organization was significantly enriched (Figure 5(e)). Among the top 15 enriched KEGG pathways, the FoxO signaling pathway, apoptosis, and PI3K-AKT signaling pathway were found (Figure 5(f)), which also existed in the KEGG pathway of network pharmacology. Bioinformatics analysis supported the positive effect of NBP in the treatment of OA. The results indicated that NBP could inhibit OA development by regulating apoptosis and PI3K/AKT/FoxO3a pathway.

### 3.8. NBP Regulated the PI3K/AKT/FoxO3a Pathway in Human OA Chondrocytes

To verify whether NBP regulated PI3K/AKT/FoxO pathway, human OA chondrocytes were treated with NBP at different concentrations (0, 0.01, 0.1, 1, and 10 *μ*M) for 24 h. Western blot analysis demonstrated that phosphorylation of PI3K and AKT significantly decreased in the NBP-treated group compared with the control group (Figure 6(a)). Moreover, NBP inhibited the protein expression of p-FoxO3a and increased accumulation of FoxO3a at the concentration of 0.01and 0.1 *μ*M, while the expression of FoxO3a was downregulated when the concentration was higher than 1 *μ*M (Figure 6(b)). The qRT-PCR result also showed that NBP significantly upregulated the level of FoxO3a at the concentration of 0.1 *μ*M (Figures 6(c)–6(e)). However, there was no remarkable effect of NBP on protein and mRNA expressions of FoxO1 and FoxO4. Immunofluorescence staining demonstrated that the expression of FoxO3a was significantly upregulated in chondrocytes after the NBP treatment (0.1 *μ*M) for 24 h (Figure 6(f)). The results demonstrated that NBP regulated the PI3K/AKT/FoxO3a pathway in human OA chondrocytes.

### 3.9. NBP Increased ECM Anabolism and Inhibited Apoptosis of Human OA Chondrocytes by Regulating FoxO3a

To identify the mechanisms of NBP on ECM anabolism and apoptosis, human OA chondrocytes were transfected with FoxO3a shRNA knockdown lentiviral particles (Lv-FoxO3a). FoxO3a knockdown lentiviral effectively decreased the FoxO3a protein and mRNA levels in chondrocytes (Figures 7(a) and 7(b)).

After chondrocytes were treated with NBP (0.1 *μ*M) and/or Lv-FoxO3a for 24 h, Lv-FoxO3a significantly downregulated the NBP-increased protein expressions of COL2A1 and ACAN (Figure 7(c)). The immunofluorescence staining of COLII was consistent with Western blot analysis (Figure 7(d)). Moreover, the NBP-increased mRNA levels of ECM-related genes (COL2A1, ACAN, SOX9, and PRG4) were significantly downregulated when chondrocytes were treated with Lv-FoxO3a for 24 h (Figure 7 E-H).

In order to determine the downstream genes in FoxO pathway after NBP treatment, chondrocytes were treated with NBP (0.1 *μ*M) and the mRNA levels of FoxO downstream genes were determined by the cluster analysis. The results showed that TNFSF10, FASL, and BCL2L11 were significantly downregulated, while BCL-6 was significantly upregulated, which were closely related to apoptosis (Figure 8(a)).

Furthermore, the mechanism of NBP on apoptosis was further investigated after chondrocytes were treated with NBP (0.1 *μ*M) and/or Lv-FoxO3a for 24 h. NBP treatment inhibited the mRNA and protein expressions of Bax and Caspase 3, while increasing expression of Bcl-2. However, the inhibitory effect of NBP on apoptosis was partially weakened after FoxO3a was transfected into chondrocytes (Figures 8(b)–8(d)). These results demonstrated that NBP increased cartilage ECM synthesis and inhibited apoptosis by upregulating FoxO3a expression in chondrocytes.

## 4. Discussion

In our present study, strong evidence demonstrated that NBP could promote cartilage ECM synthesis and inhibit OA development. NBP promoted ECM anabolism in human OA chondrocytes and cartilage explants and inhibited the apoptosis and oxidative stress of chondrocyte. Moreover, NBP inhibited the development of knee OA in the DMM+ACLT rat model. Bioinformatics analysis using network pharmacology and transcriptome sequencing were performed to explore the mechanism of NBP on inhibiting OA development. The results showed that NBP could regulate PI3K/AKT/FoxO pathways and inhibit chondrocyte apoptosis. Further analysis indicated that NBP regulated FoxO3a expression in chondrocytes mainly through PI3K/AKT pathway in vitro. Interestingly, we found that in FoxO3a knockdown chondrocytes not only the effect of NBP on promoting the formation of extracellular matrix components was attenuated but also the inhibitory effect of NBP on chondrocyte apoptosis was also weakened. Therefore, NBP may be a potential therapeutic drug for OA (Figure 9).

As the only cell type in the cartilage, chondrocytes have a vital effect in maintain the structure and function of cartilage. Degeneration of cartilage is generally accompanied by excessive apoptosis of chondrocytes [22]. The degree of apoptosis is closely related to the severity of cartilage damage and matrix degradation, indicating that apoptosis plays an important role in the pathogenesis of OA [5, 23]. Oxidative stress is also a potential mechanism of OA degeneration [24]. Excessive oxidative stress resulted in the accumulation of ROS (superoxide anion and peroxides), but the ROS scavenging enzymes including SOD, GSH, and CAT failed to eliminate ROS [25]. Excessive oxidative stress could lead to apoptosis of chondrocytes and cartilage destruction [26]. Our study showed that NBP promoted cartilage ECM synthesis and inhibited the development of knee OA in rat model. Moreover, flow cytometry and TUNEL staining showed that NBP downregulated the chondrocyte apoptosis and western blot analysis also demonstrated that NBP inhibited the expressions of apoptotic-related proteins and ROS scavenging enzymes, indicating that NBP could inhibit apoptosis and oxidative stress in human OA chondrocytes.

Bioinformatics is one of the effective ways to definite the mechanism of drug action. We combined network pharmacology with transcriptomics and identified common signaling pathways PI3K/AKT and FoxO. FoxO is a downstream target of PI3K/AKT pathway that is closely related to cell proliferation, cell apoptosis, autophagy, and antioxidant activity [27]. FoxO transcription factors are negatively regulated by AKT-mediated phosphorylation [28]. AKT can facilitate the phosphorylation of FoxO by inducing the binding of FoxO to 14-3-3 protein, which promotes the translocation of FoxO1, FoxO3, and FoxO4 from the nucleus to the cytoplasm. Meanwhile, the prevention of relocation to the nucleus can inhibit the transcription of FoxO [29–31]. Akasaki et al. reported that FoxO was predominantly located in the chondrocyte cytoplasm in OA cartilage, whereas it was predominantly in the nucleus in normal cartilage [32]. In our study, the expression levels of p-PI3K and p-AKT were downregulated after human OA chondrocytes were treated by NBP, while the expression of FoxO3a was upregulated. As indicated by the results, NBP inhibited PI3K/AKT, thus reducing the inhibition of AKT on FoxO3a and weakening the phosphorylation of FoxO3a, which facilitated the nuclear localization of FoxO3a.

FoxO transcription factors were the central regulators of cellular homeostasis. In humans, the FoxO family consists of FoxO1, FoxO3a, FoxO4, and FoxO6. FoxO transcription factors could regulate various cellular processes, including cell cycle regulation, redox balance, autophagy, apoptosis, metabolism, and repair of DNA damage [29, 33, 34]. FoxO is an important regulator of cartilage homeostasis and involved in the formation, development, and maturation of cartilage [35, 36]. Akasaki et al. found the various expressions of FoxO in the cartilage of mice of different ages and different months [32]. Matsuzaki et al. reported that FoxO promoted the expression of PRG4 and confirmed downregulated FoxO expression in aging and OA cartilage, while the absence of FoxO3 results in more severe OA with an earlier occurrence, indicating that maintenance or restoration of FoxO expression could delay OA progression [37]. Interesting, the protein encoded by FoxO1 and FoxO3 is highly expressed in a normal human cartilage, while FoxO4 expression is much lower [38].

Our results showed that the expression of FoxO3a significantly increased and the expression of p-FoxO3a declined after NBP treatment, while there was no significant difference in the expressions of FoxO1 and FoxO4. Moreover, it was found that the increased expressions of ECM components such as COL2A1, ACAN, SOX9, and PRG4 after NBP treatment significantly decreased after the knockdown of FoxO3a. Therefore, the results demonstrated that NBP may have an effect on ECM composition by regulating FoxO3a expression.

As a transcription factor, FoxO3a can regulate the apoptosis of various cells [39, 40]. Zou et al. showed that FoxO3a mediates TRIM33 regulation of oxidative stress-induced apoptosis in osteoblasts, suggesting FoxO3a could inhibit osteoblast apoptosis [13]. In this study, cluster analysis based on the mRNA levels of downstream genes of FoxO indicated that numerous apoptosis-related genes were significantly changed. In the present study, NBP could inhibit chondrocytes apoptosis, but the inhibitory effect of NBP on apoptosis was significantly attenuated after knockdown of FoxO3a in human OA chondrocytes. Therefore, we conclude that FoxO3a may be involved in NBP-inhibited apoptosis of human OA chondrocytes.

It is worth noting that the behavior of cells is determined by a variety of signal pathways and different regulatory mechanisms, which are complex and interactive [41]. The limitation of our study is that the therapeutic effect of NBP on OA and its mechanism are still in the preliminary exploration stage, and other potential mechanisms (such as inflammation and autophagy) have not been further explored. Thus, we will further explore the detailed effect and mechanism of NBP on promoting chondrocyte survival and inhibiting OA development in the future.

## 5. Conclusions

In conclusion, our study demonstrated NBP could promote the expression of FoxO3a by regulating the PI3K/AKT pathway, which further inhibited chondrocyte apoptosis. Through the above pathways, NBP facilitated the production of ECM components in chondrocytes and inhibited osteoarthritis development in rats. These findings confirmed that NBP was a potential drug in promoting cartilage ECM synthesis and provided some guidance for the treatment of clinical OA.

## Figures and Tables

**Figure 1:** NBP was identified as a chondrogenic inducer that increased ECM anabolism of human OA chondrocytes in vitro. (a) Chemical structure of NBP. (b) Alcian blue staining (scale bar, 100 *μ*m). (c) Immunofluorescence staining of COLII (scale bar, 100 *μ*m). (d) The CCK8 assay measured the cytotoxicity of NBP on chondrocytes at different concentrations for 24 h. (e, f) The protein expressions of COL2A1 and ACAN were detection by Western blot analysis after chondrocytes were treated with NBP for 24 h. (g) The mRNA levels of COL2A1, ACAN, PRG4, and SOX9 were detected using qRT-PCR. (h, i) The expressions of COLII and ACAN were detected by the immunofluorescence assay (scale bar, 100 *μ*m). All data are expressed as the mean ± standard deviation (SD). ^∗^*P* < 0.05,  ^∗∗^*P* < 0.01, and^∗∗∗^*P* < 0.001.

**Figure 2:** NBP promoted ECM anabolism in OA cartilage explants. (a) Proteoglycan content was measured by the safranin O-fast green staining after incubation with NBP for 2 w (scale bar, 100 *μ*m). (b) COLII content was measured by immunohistochemistry staining (scale bar, 100 *μ*m). (c) Average optical density values of proteoglycan content determined by safranin O-fast green staining. (d, e) GAG and DNA content per wet weight were assessed after NBP (0.1 *μ*M) treatment for 2 w. (f–i) The mRNA levels of COL2A1, ACAN, PRG4, and SOX9 were detected using qRT-PCR after NBP (0.1 *μ*M) treatment for 2 w. All data are expressed as the mean ± standard deviation (SD). ^∗^*P* < 0.05,  ^∗∗^*P* < 0.01, and^∗∗∗^*P* < 0.001.

**Figure 3:** NBP inhibited the development of knee OA after intra-articular injection of NBP in a rat model of DMM+ACLT for 8 w. (a) Representative images of HE for cartilage destruction, safranin O-fast green for cartilage regeneration, and immunohistochemistry staining for COLII expression, respectively. (b) OARSI scores in different treatment groups (*n* = 6). (c) Pain response time when rats were placed onto a 55°C hot plate after the surgery (*n* = 6). (d) The differences in two hind limb weights after the surgery in rats (*n* = 6). All data are expressed as the mean ± standard deviation (SD). ^∗^*P* < 0.05,  ^∗∗^*P* < 0.01, and^∗∗∗^*P* < 0.001.

**Figure 4:** NBP inhibited apoptosis and oxidative stress of human OA chondrocytes. (a, c) Apoptosis was analyzed by flow cytometry and apoptosis rates are expressed in the respective group. (b, d) Apoptotic assay by TUNEL staining was observed under a microscope, and TUNEL-positive cells were calculated (*n* = 3, scale bar, 100 *μ*m). (e, f) The mRNA levels of Bcl-2 and Bax were measured by qRT-PCR. (g) The protein expressions of CAT, SOD2, Bcl-2, Bax, and Caspase 3 were determined after treatment with NBP (0-10 *μ*M) for 24 h by Western blot analysis. (h, i) The expression levels of SOD and GSH in chondrocytes treated with NBP (0-10 *μ*M) for 24 h. (j, k) The mRNA levels of SOD2 and CAT were measured by qRT-PCR. All data are expressed as the mean ± standard deviation (SD). ^∗^*P* < 0.05,  ^∗∗^*P* < 0.01, and^∗∗∗^*P* < 0.001.

**Figure 5:** Bioinformatics analysis based on network pharmacology and transcriptome sequencing result after treated with NBP. (a–c) Network pharmacology. (a) Venn diagram of NBP-OA. (b) Bubble plot of the enrichment analysis results: cell components. (c) Signaling pathways. (d–f) Transcriptome sequencing. (d) Volcano plots of differentially expressed genes in the transcriptome. (e) Gene Ontology (GO) analysis of the transcriptome of chondrocytes administrated with NBP. (f) Pathway analysis from the chondrocyte transcriptome.

**Figure 6:** NBP regulated the PI3K/AKT/FoxO3a pathway in human OA chondrocytes. (a, b) The protein expressions of FoxO1, FoxO3a, p-FoxO3a, FoxO4, PI3K, p-PI3K, AKT, and p-AKT were determined by Western blot assay. (c–e) The mRNA levels of FoxO1, FoxO3a, and FoxO4 were measured using qRT-PCR. (f) Immunofluorescence staining of FoxO3a and ACTIN (scale bar, 20 *μ*m). All data are expressed as the mean ± standard deviation (SD). ^∗^*P* < 0.05,  ^∗∗^*P* < 0.01, and^∗∗∗^*P* < 0.001.

**Figure 7:** NBP increases ECM anabolism in human OA chondrocytes by regulating FoxO3a. (a, b) The protein and mRNA levels of FoxO3a were evaluated by Western blot and qRT-PCR after treated with and/or Lv-FoxO3a for 24 h. (c) Proteins expressions of ACAN and COL2A1 were detected by Western blot. (d) Immunofluorescence staining for COLII (scale bar, 50 *μ*m). (e–h) The mRNA levels of COL2A1, ACAN, SOX9, and PRG4 were determined by qRT-PCR. All data are expressed as the mean ± standard deviation (SD). ^∗^*P* < 0.05,  ^∗∗^*P* < 0.01, and^∗∗∗^*P* < 0.001.

**Figure 8:** NBP inhibited apoptosis of human OA chondrocytes by upregulating FoxO3a. (a) Cluster analysis of mRNA levels of downstream genes in the FoxO pathway. (b, c) The mRNA levels Bcl-2 and Bax were determined. (d) The protein expressions of Bcl-2, Bax, and Caspase 3 were determined. All data are expressed as the mean ± standard deviation (SD). ^∗^*P* < 0.05,  ^∗∗^*P* < 0.01, and^∗∗∗^*P* < 0.001.

**Figure 9:** Molecular mechanism of NBP on inhibiting OA development. NBP possesses protective effect on human OA chondrocytes from apoptosis by regulating PI3K/AKT/FoxO3a pathway (created with https://biorender.com/).

**Table 1:** Sequences of primers used for real-time PCR.

Genes	Primer sequence (5′-3′)
COL2A1	S: 5′-GATGCCACACTCAAGTCCCTCA-3′
	A: 5′-TGCTGCTCCACCAGTTCTTCTT-3′
ACAN	S: 5′-CACTGTTACCGCCACTTCCC-3′
	A: 5′-CATCATTCCACTCGCCCTTCT-3′
SOX-9	S: 5′-GTCAACGGCTCCAGCAAGAA-3′
	A: 5′-CGTTCTTCACCGACTTCCTCC-3′
PRG4	S: 5′-TCCATTCAGTCCACCATCTCC-3′
	A: 5′-ACTGCTGAATGCTGCCACCT-3′
Bax	S: 5′-CGGGTTGTCGCCCTTTTCTA-3′
	A: 5′-GAGGAAGTCCAATGTCCAGCC-3′
Bcl-2	S: 5′-GGAGGATTGTGGCCTTCTTTG-3′
	A: 5′-GCATCCCAGCCTCCGTTATC-3′
SOD2	S: 5′-GGGACACTTACAAATTGCTGCTT-3′
	A: 5′-CATTCTCCCAGTTGATTACATTCC-3′
CAT	S: 5′-TCGGTTCTCCACTGTTGCTG-3′
	A: 5′-ACGTAGGCTCCAGAAGTCCCA-3′
FoxO1	S: 5′-CTCACCCATTATGACCGAACAG-3′
	A: 5′-TTTGGTAGTTTGGGCTGGGT-3′
FoxO3a	S: 5′-CGGACAAACGGCTCACTCT-3′
	A: 5′-GCTCTTGCCAGTTCCCTCATT-3′
FoxO4	S: 5′-TCAGCAGGATGGAAGAACTCG-3′
	A: 5′-CTGGCAGCACAGATGGTTTC-3′
GAPDH	S: 5′-GGAAGCTTGTCATCAATGGAAATC-3′
	A: 5′-TGATGACCCTTTTGGCTCCC-3′

S: sense; AS: antisense.

## Data Availability

All data during the study are available from the corresponding authors by request.
